The article "Quality of Sleep in an HIV Population on Antiretroviral Therapy at an Urban Tertiary Centre in Lagos, Nigeria" was published in 2014. Journal: Neurol Res Int.

# Quality of Sleep in an HIV Population on Antiretroviral Therapy at an Urban Tertiary Centre in Lagos, Nigeria

**DOI:** 10.1155/2014/298703

**Published:** 2014-04-28

**Authors:** Olajumoke Oshinaike, Akinsegun Akinbami, Olaitan Ojelabi, Akinola Dada, Adedoyin Dosunmu, Sarah John Olabode

**Affiliations:** ^1^Department of Medicine, Lagos State University College of Medicine, Lagos, Nigeria; ^2^Department of Haematology and Blood Transfusion, Lagos State University College of Medicine, Lagos, Nigeria; ^3^Department of Hematology, Ben Carson College of Medicine, Babcock University, Ogun, Nigeria

## Abstract

*Aim*. To determine the prevalence of sleep disturbance and its associated characteristics in HIV-positive outpatients on HAART using the PSQI. *Methods*. Using a cross-sectional design, 300 patients attending the outpatient HIV/AIDS clinic at the Lagos State University Teaching Hospital were recruited. Baseline data obtained included the participants' demographic data, educational qualification, and marital status. Their treatment history, including duration since HIV diagnosis, the most recent CD4 cell count, and current antiretroviral therapies, was obtained from their case records. Each participant completed the PSQI questionnaire and those with scores ≥5 were diagnosed with poor sleep quality. *Results*. The participants were made up of 70.7% females and 29.3% males. Their ages ranged between 18 and 74 years with a mean of 38.9 ± 10.3 years. According to the PSQI, 59.3% reported poor sleep quality. The mean score of those with poor quality sleep (9.2 ± 3.3) was comparable to that of those with good quality sleep (1.26 ± 1.4). *P* < 0.001. Significant differences were observed in all the individual components of the PSQI (*P* < 0.001). On multivariate analyses, the independent associations with sleep quality were the duration since HIV diagnosis (*P* = 0.29), efavirenz based regimen (*P* < 0.001), and lower CD4 cell count (*P* < 0.001). *Conclusions*. Sleep disturbances are quite common in the HIV population even in the era of HAART. Early recognition via routine assessment and effective treatments could prevent the resultant complications and improve quality of life.

## 1. Introduction

Sleep is a natural process that restores body functions including immune system health. Sleep disturbances can interfere with normal physical, mental, and emotional functioning and have been reported in HIV-infected individuals since the 1980's [1–4]. HIV-infected individuals have been known to have a high prevalence of sleep disturbance, between 40 and 70% [5–7].

Both effects of the virus and antiretroviral drugs may cause sleep disturbances. Earlier studies have reported high rates of neuropsychiatric side effects including insomnia in patients on efavirenz based therapies. Efavirenz is known to increase sleep latency and decrease sleep duration with symptoms resolving usually within the first weeks of treatment [8, 9]. Most CNS symptoms of efavirenz including insomnia are mild but some patients change therapy because of unbearable neurotoxicity. Other clinical studies have reported increased serum levels of efavirenz and higher rates of neuropsychiatric disorders in patients of African origin [10, 11]. It is thought that the defective* CYP2B6 G516T* variant allele which is common in African population impairs efavirenz metabolism, thus increasing efavirenz plasma concentrations, thereby leading to toxicity [12, 13]. The burning pain of peripheral neuropathy [14] and night sweats can also interrupt sleep. Other psychosocial causes of sleep disturbances in the HIV population include anxiety over the illness, financial concerns, stigmatization, depression, suicidal thoughts, and unemployment.

Sleep disturbances occur throughout the stages of infection, being more prevalent in the advanced stage [15, 16]. It can lead to impairment of attention, concentration, fatigue, memory, mood swings, and reduction in energy levels [17, 18]. It may also increase the risk for psychiatric disorders, cardiovascular morbidity, and mortality and health care utilization [18–21].

Results from recent studies have shown that HIV individuals with sleep problems are less likely to adhere to their antiretroviral therapy regimens probably as a result of depression [22–24]. Nonadherence may result in treatment failure, disease progression, and the development of resistant strains [25, 26]. Sleep disorders in HIV population are treatable with early therapy effectively lowering the risk of these complications. Management includes the use of pharmacologic agents such as benzodiazepines, nonbenzodiazepine hypnotics, and antidepressants and psychological and behavioural treatments such as cognitive behavioural therapy and improved sleep hygiene.

With the increasing life expectancy in HIV individuals, sleep disturbances may adversely impact on their quality of life and work performance. Determining the quality of sleep and its effects could prevent resultant complications that may arise. We aimed to determine the quality of sleep and its associated factors including efavirenz based therapies in our African population of HIV-positive individuals.

## 2. Methodology

### 2.1. Study Design and Participants

This is a cross-sectional study conducted at the HIV clinic of the Lagos State University Teaching Hospital (LASUTH) between January and September 2013. The study enrolled patients attending the HIV clinic, who were at least 18 years, diagnosed with HIV infection, on antiretroviral therapy, not working nightshift schedules, and not pregnant within the prior 3 months. Exclusion criteria included recent use of hard/illicit drugs or alcohol, depression, current or recent suicidal ideation, and the presence of any acute medical condition that could affect the participant's sleep, cognitive function, or ability to complete the study questionnaire. The hospital ethics committee approved this research, and each participant gave informed consent.

### 2.2. Methods

After signing informed consent, information regarding the participant's demographic data, educational qualification, and marital status was obtained and documented. Their treatment history, including duration of HIV diagnosis, the most recent laboratory results for CD4 cell count, and current antiretroviral therapy, was also obtained from their case records.

### 2.3. Subjective Sleep Assessment

Each participant was administered the PSQI, a 19-item questionnaire that assesses sleep components including sleep quality, sleep latency, sleep duration, habitual sleep efficiency, sleep disturbances, use of hypnotics, and daytime dysfunction during the last month. The PSQI has been used and validated in different settings for the measurement of quality and pattern of sleep in adults. Each individual component receives a score from zero to three, with the final score on the instrument ranging between 0 and 21. The higher the score, the worse the quality of sleep, and scores ≥5 indicate poor sleep quality [27].

### 2.4. Data Analysis

Data were analysed using SPSS version 19.0 statistical package. Continuous variables such as participant's age, HIV diagnosis duration, CD4 cell count, and PSQI score are presented as mean ± standard deviation (SD) and comparison between groups was made using multivariate logistic regression analysis. Categorical variables (e.g., gender, marital status category, HAART group category, and CD4 cell count category below or above 200 cells/mm^3^) are presented as frequencies (%) and group differences compared using nonparametric Yates corrected *X* ^2^ test. The level of significance was considered as <0.05.

## 3. Results

### 3.1. Demographic and Clinical Characteristics of Study Participants

The characteristics of the 300 participants included in this analysis are summarized in Table 1. The sample was predominantly female and all were on antiretroviral therapy, with a mean duration of 27.5 ± 33.3 months at the time of the study.

### 3.2. Sleep Quality Assessment

According to the PSQI, 40.7% patients reported having good sleep quality, whereas 59.3% reported poor sleep quality. Those with good sleep quality were 42 males and 80 females with ages ranging between 25 and 70 years (mean 39.1 ± 9.4) whilst those with poor quality sleep were 46 males and 132 females with ages ranging between 18 and 74 years (mean 38.7 ± 10.9); *P* = 0.78. The PSQI scores of those with poor quality sleep ranged between 5 and 19 with a mean of 9.2 ± 3.3 (median 9.0; range 14) whilst that of those with good quality sleep ranged between 0 and 4 with a mean of 1.26 ± 1.4 (median 1.0; range 4); *P* < 0.001. The characteristics that showed a significant association with the participants' quality of sleep are listed in Table 2. Age, gender, educational qualification, and marital status were not significantly associated with the quality of sleep. The relationship between each of the significant correlates (duration since HIV diagnosis, efavirenz based regimen, and lower CD4 cell count) and sleep quality was further examined using multivariate logistic regression models (Table 3). The individual component scores of the PSQI were compared in patients with good and poor quality sleep in Table 4. Significant differences were observed in all the individual components (*P* < 0.001).

## 4. Discussion

In this study, using the PSQI questionnaire, we assessed sleep quality in our outpatients HIV cohort over the last month and observed that 59.3% of cases had poor quality sleep. This rate is high and in the range of that documented in comparable studies that have assessed sleep quality using the PSQI. Crum-Cianflone et al. and Ferreirra and Ceolm had documented slightly lower rates of 46.7% and 46%, respectively [28, 29]. Our rate is however lower than the 73% documented by Rubinstein et al. probably as a result of our exclusion criteria. We had excluded cases with the use of hard drugs and alcohol, depression, and suicidal ideation from our study. Varying prevalent rates of sleep disturbances in people living with HIV have been documented in literature probably as a result of the difference in the diagnostic criteria of sleep disturbances [30, 31]. Our findings are however similar to those in other studies that have documented high rates of sleep disturbances in the era of HAART [32, 33]. It is worthy to note that our HIV population live in a highly urbanized area where other causes of sleep disturbances exist. Lagos state with its high population, high level of night time social activities, and night time road traffic noise pollution may be contributory to this high prevalence. Studies have shown that urban population living in noisy areas have a higher risk of sleep disturbances [34].

The mean total PSQI score in the cases with poor quality sleep in our study was 9.2. This is in the range of that found in other studies. Nokes and Kendrew and Hand et al. had documented similar scores of 10.0 and 12.3, respectively, in their cohorts [35, 36]. We also noted a significant difference in all the components of sleep quality assessed in poor sleepers compared with those with good quality sleep. This finding has also been documented in earlier studies [29, 37]. Sleep architecture in HIV patients is characterised by increased sleep latencies, frequent nocturnal awakenings, a reduction in the hours of sleep, early morning awakening with a reversal of the slow wave sleep, and rapid eye movement sleep patterns.

All these are thought to be as a result of underlying immune dysfunction. Though the regulation of cytokines in the brain is complex, it is known that some cytokine-associated substances, such as the IL1RA and the TNF and IL1 soluble receptors, act as endogenous antagonists, inhibiting spontaneous sleep [38]. Also elevated levels of ILs 2, 4, 6, 8, 10, 13, and 18; IFNs *α*, *β*, and *γ*; and transforming growth factor cause a decrease in NREM sleep [39, 40]. Growth hormone dysregulation together with the physiologic coupling that has been demonstrated between alpha tumor necrosis factor and delta wave amplitude may also contribute to this sleep pathology.

There have been inconsistent reports on the relationship between CD4 cell count and poor sleep quality. Some studies [35, 41, 42] have not found any relationship whilst others have confirmed that sleep disturbances are independently related to immune status [37, 43, 44]. We noted a significant association between poor quality sleep and lower mean CD4 count in our study. Research has shown that the immune system is directly linked to the psyche by a complex network of nerves, hormones, and neuropeptides. This network of specific physiological pathways allows immune function to have a direct impact on health especially sleep.

We noted that a significant proportion of patients on efavirenz based HAART therapy had poor quality sleep. Other earlier studies had also documented a correlation between high blood concentrations of efavirenz and poor sleep pattern [44, 45]. Gallego et al. had performed ambulatory electroencephalogram monitoring on HIV-infected subjects treated with efavirenz and found that those receiving efavirenz had longer sleep latencies and shorter duration of deep sleep. Also, efavirenz plasma levels were significantly higher in patients with insomnia and/or reduced sleep efficiency [46]. It had been suggested that a direct inhibition of serotonergic hypothalamic pathways by efavirenz may explain this.

This may also be attributed to the presence of the defective* CYP2B6 G516T* variant allele known to be common in black Africans, in our cohort. This genetic abnormality causes a variation in the rate of efavirenz metabolism thereby significantly increasing the likelihood of the occurrence of sleep disturbance.

In our study, the length of time from HIV diagnosis was found to be associated with sleep disturbances, with a significant association between shorter duration from diagnosis and poor quality of sleep. HIV infection is a highly stigmatized illness with a sense of dejection and loss of self-esteem, all symptoms of depression and normal emotional responses to the reality of living with HIV. These may explain the higher rate of sleep disturbances in the months, soon after diagnosis. This finding however is conflicting with that of other studies that have assessed sleep disturbances in relation to duration of infection. Imeri and Opp and Seay et al. did not document any association in their studies [40, 44].

## 5. Conclusion

The results of this study indicate that sleep disturbances are quite common in people living with HIV infection in this population with an anticipated negative impact on the quality of life. Early recognition via routine assessment and implementation of effective medical and behavioural treatments could improve functioning and reduce complications. Future studies are required to determine the frequency of the genetic polymorphism affecting efavirenz metabolism in the African population. Also the regions in Africa where this defective gene exists need to be defined. More studies need to be conducted to determine if the genetic testing can help individualize therapy, avoid toxicity, and maximize efficacy. Treatment guidelines for proper management of sleep disturbances in the HIV population need to be designed whilst taking into consideration drug interactions.

## Figures and Tables

**Table 1:** Demographic and clinical characteristics of study population.

Variable	*N* = 300 (%)
Age, Mean (SD) years	38.9 ± 10.3
Gender	
** **Male	88 (29.3)
Female	212 (70.7)
Education	
** **None	17 (5.7)
Primary	73 (24.3)
Secondary	135 (45)
Tertiary	75 (25)
Marital status	
** **Married	224 (74.7)
Single	55 (18.3)
Widowed	15 (5)
Divorced	4 (1.3)
Separated	2 (0.6)
CD4 count, Mean (SD) cells/mm^3^	334.2 ± 215.4
Cd4 ≤ 200	97 (32.3)
Cd4 > 200	203 (67.7)
HAART type	
** **Efavirez based	62 (20.7)
Non efavirez based	238 (79.3)
HIV diagnosis duration, Mean (SD) months	27.5 + 33.3

**Table 2:** Demographic and clinical characteristics of patients with poor and good quality sleep.

Variables	Poor quality sleep (*n* = 178)	Good quality sleep (*n* = 122)	*P* value
Age, Mean (SD) years	38.7 (±10.9)	39.1 (±9.4)	NS
Sex			
Male	46 (25.8%)	42 (34.4%)	NS
Female	132 (74.2%)	80 (65.6%)	
Marital status			
Single/separated/widowed	51 (28.7%)	25 (20.5%)	NS
Married	127 (71.3%)	97 (79.5%)	
Duration of HIV diagnosis,	23.7 (±28.6)	32.9 (±38.5)	0.018
Mean (SD) months			
≥Secondary education	118 (66.3%)	92 (75.4%)	NS
<Primary/Nil education	58 (32.6%)	32 (26.2%)	
HAART type			
Efavirenz based	54 (30.3%)	8 (6.5%)	<0.001
Non efavirenz based	124 (69.6%)	114 (93.4%)	
CD4 count			
≤200	77 (43.3%)	20 (16.4%)	<0.001
>200	101 (56.7%)	102 (83.6%)	
Mean CD4 count (SD)	293.1 (±197.7)	392.6 (±226.4)	<0.001
Mean PSQI score (SD)	9.21 (±3.3)	1.30 (±1.4)	<0.001

NS: Not significant.

**Table 3:** Relationship of the significant correlates with sleep quality using multivariate logistic regression.

Variable	*B*	Standard error	*P* value
HAART type	1.466	0.378	<0.001
(Efavirenz/non efavirenz based)			
HIV diagnosis duration	0.269	0.256	0.293
(</>12 months)			
CD4 category	1.201	0.295	<0.001
(≤ or >200)			

**Table 4:** Comparison of the individual component score of the PSQI amongst patients with poor and good quality sleep.

PSQI components	Poor quality sleep	Good quality sleep	*P* value
	Mean (SD)	Mean (SD)	
C-1 Quality of sleep	1.63 ± 0.71	0.21 ± 0.42	<0.001
C-2 Sleep latency	1.63 ± 0.76	0.27 ± 0.46	<0.001
C-3 Sleep duration	1.68 ± 0.76	0.39 ± 0.49	<0.001
C-4 Sleep efficiency	1.45 ± 0.77	0.23 ± 0.42	<0.001
C-5 Sleep disturbances	1.14 ± 0.74	0.14 ± 0.35	<0.001
C-6 Sleep medication	0.83 ± 0.66	0.02 ± 0.15	<0.001
C-7 Daytime sleepiness	0.77 ± 0.64	0.02 ± 0.12	<0.001
